RETRACTED

# Severe Acute Respiratory Syndrome Coronavirus 2 (SARS-CoV-2) Infection Mimicking as Pulmonary Tuberculosis in an Inmate

**DOI:** 10.7759/cureus.8464

**Published:** 2020-06-05

**Authors:** Hina Akbar, Rehan Kahloon, Sobia Akbar, Arslan Kahloon

**Affiliations:** 1 Internal Medicine, University of Tennessee Health Science Center, Memphis, USA; 2 Internal Medicine, Regional One Hospital, Memphis, USA; 3 Cardiology, Erlanger Health System/University of Tennessee College of Medicine, Chattanooga, USA; 4 Internal Medicine, Postgraduate Medical Institute, Lahore, PAK; 5 Gastroenterology, Erlanger Health System/University of Tennessee College of Medicine, Chattanooga, USA

**Keywords:** sars-cov-2 (severe acute respiratory syndrome coronavirus -2), pulmonary tuberculosis, inmate population, vulnerable group, prison health

## Abstract

Coronavirus disease 2019 (COVID-19) is an emerging global infectious disease with emerging medical knowledge. Clinical presentation of severe acute respiratory syndrome coronavirus 2 (SARS-CoV-2) is very variable amongst patients, and the literature about unusual presentations is growing rapidly. This lack of knowledge leads to diagnostic, therapeutic, and management challenges in such patients. Here, we describe a case of SARS-CoV-2 infection in a low prevalence area which was initially diagnosed and managed as pulmonary tuberculosis (TB) in a high-risk inmate population. These ambiguous presentations can lead to mismanagement of such patients resulting in potentially fatal outcomes and public health crises in confined facilities. This also highlights the significance of a high index of clinical suspicion for SARS-CoV-2 especially in high risk and vulnerable populations.

## Introduction

Tuberculosis (TB) and Coronavirus disease 2019 (COVID-19) also known as severe acute respiratory syndrome coronavirus 2 (SARS-CoV-2) are both infectious diseases that primarily involve the respiratory tract and the lungs. Both diseases have very similar symptoms such as cough, fever, and difficulty in breathing which could lead to significant delays in the timely diagnosis of rapidly progressing SARS-CoV-2 infection during times of the ongoing COVID-19 global pandemic. TB, however, has a longer incubation period with a slower onset of disease, whereas, symptoms onset in SARS-CoV-2 could range from asymptomatic to rapid progression but both can vary significantly over time.

SARS-CoV-2 is a novel infection and the knowledge about unusual presentations are rapidly emerging. The most commonly documented reason for hospitalization is generally respiratory distress and new onset cough which is also one of the main symptoms of pulmonary TB [1]. Newly discovered atypical features of the SARS-CoV-2 infection continue to be frequently reported, while increasing clinician’s awareness and mindfulness for uncommon or confounding presentations [1,2]. Here, we describe a case of an inmate patient considered vulnerable and at high risk for TB who was eventually diagnosed with SARS-CoV-2 infection presenting with hemoptysis.

RETRACTED

## Case presentation

A 19-year-old man who is an inmate in a local county jail was admitted to the hospital with progressive cough of two weeks duration and development of hemoptysis. The patient reported cough that was mostly dry except for frequent episodes of hemoptysis recently. He denied any fever, nausea, vomiting, or diarrhea. He did complain of mild malaise and intermittent right-sided chest pain on deep inspiration. He reported 10 pounds of weight loss and a decreased appetite over the last several months. He reported his cellmate of many months was recently diagnosed with TB. He had a skin purified protein derivative (PPD) test placed in prison facility which showed active induration of 12 mm suggesting TB infection. Social history was negative for smoking and he has been incarcerated for the last six months; he was living with the same cellmate. Upon concerns of pulmonary TB with worsening hemoptysis, he was sent to a tertiary hospital for management.

On presentation, he was in no respiratory distress with 15 breaths per minute and oxygen saturation of 98% while breathing ambient air. His respiratory exam was unremarkable with clear to auscultate lungs without wheezing or crackles. Laboratory studies were notable for mild lymphopenia (3.4 cells/L) with 44% lymphocytes. He had elevated lactate dehydrogenase (331 U/L), D-Dimer (0.54), and a normal ferritin and C-reactive protein levels. Chest X-ray did not reveal any infiltrates or effusions (Figure 1). 

**Figure 1:** Chest X-ray Chest X-ray showing increased hilar hypervascularity due to inflammation. No distinct infiltrates seen.

Considering the high risk history of TB exposure while in the prison cell and with suggestive PPD results, the patient was thought to have pulmonary TB. A CT scan of the chest performed for further work up of hemoptysis and weight loss revealed enlarged left hilar lymph node confluence and four small pleural based pulmonary nodules in the left lung with the largest measuring 1.8 cm (Figure 2).

**Figure 2:** CT scan of the chest Arrow in blue showing hilar lymphadenopathy. Arrow in orange showing pleural nodules.

The appearance was noted to be compatible with mycobacterial infection. 

The patient was placed in respiratory isolation and further work up for TB was started. Further testing with QuantiFERON-TB Gold test was negative. He also had three samples of sputum acid-fast bacillus (AFB) smear and culture that came back negative. This raised suspicion if the patient had another respiratory illness which was mimicking as TB.

RETRACTED

Patient was then tested for SARS-CoV-2 and COVID-19 infection was eventually confirmed by a real time reverse-transcription-polymerase chain-reaction assay. He was subsequently placed in airborne and contact/droplet isolation and manged for COVID-19 viral infection with symptomatic treatment and antiviral therapy according to the guidelines and management for COVID-19. The hemoptysis gradually decreased and the patient gradually recovered after being in the hospital for ten days.

## Discussion

The SARS-CoV-2 pandemic is challenging and, in many cases, an overwhelming situation for the medical community as new knowledge is reported every day. Data regarding variable and multitude of clinical presentations related to this novel coronavirus is rapidly growing as new cases of SARS-CoV-2 are being reported from across different regions and communities like prisons. The list of common symptoms like fever (88% of cases), cough (68%), vomiting (5%), and diarrhea (3.8%) is growing as newer data becomes available [1-3]. Although fever and respiratory symptoms are typical hallmarks of COVID-19 infection, other acute signs and symptoms should not be ignored during this pandemic era. Hemoptysis has been rarely reported in patients with COVID-19 infections to date as manifested by our patient [3-6]. Furthermore, subtle findings of hilar lymphadenopathy on CT imaging, as seen in our patient, can be another clue in such patients [7-9]. 

Currently, most public health measures to control the spread of COVID-19 rely heavily on the identification of individuals with the highest probability of COVID-19. To identify such individuals the World Health Organization (WHO) has developed case definitions for testing [5], which rely on both the presence of classical symptoms and the epidemiological risk [2,5]. However, these definitions do not capture infected individuals with atypical presentations.

The patient described in this report highlights an atypical host response to SARS-CoV-2, as hemoptysis is not included in the current suspected COVID-19 case definition criteria based on epidemiological exposure. Similar reports as ours were reported from China and South Korea as reported by Shi et al. [10]. Our patient also presented with hemoptysis after roughly two weeks of non-specific symptoms and the first consideration was of TB upon admission. 

Failing to identify all infected individuals within a healthcare facility increases the risk of virus transmission within the facility and places both healthcare workers and other patients at risk of infection [6]. In addition, the failure to properly diagnosis COVID-19 hinders the provision of appropriate care. 

RETRACTED

Our case further highlights the importance of picking such infections early on in confined facilities like prisons and nursing homes where infection can spread rapidly in otherwise vulnerable populations. This poses a significant public health problem considering the complexity of resources required to control spread in such facilities [11,12]. Citizens held in prisons and other detention facilities also need to be considered as part of the broader public health response to COVID-19.

## Conclusions

This case highlights a unique presentation of COVID-19 in the prison population. Cases of SARS-CoV-2 continue to emerge with atypical presentations such as the case highlighted here. The recognition of this atypical presentation and utilization of a more liberal testing strategy even in asymptomatic, and especially for at-risk populations (e.g., inmates, nursing homes), is crucial to the avoidance of outbreaks of pandemic diseases in such facilities. Therefore, it is important for all physicians and particularly, the staff of prison facilities to have a high clinical suspicion for SARS-CoV-2 to prevent outbreaks in confined facilities.
